The article "Physical Education Teaching Strategy under Internet of Things Data Computing Intelligence Analysis" was retracted in 2023. Reasons: suspected computer-generated content; unreliable results or conclusions; lack of ethics approval or compliance; missing or withdrawn patient consent.

# Physical Education Teaching Strategy under Internet of Things Data Computing Intelligence Analysis

**DOI:** 10.1155/2022/5299497

**Published:** 2022-04-11

**Authors:** Pingting Zhang, JianPeng Hou

**Affiliations:** Sports Teaching and Research Department, Heilongjiang University, Harbin 150040, Heilongjiang, China

## Abstract

Racket sports such as tennis are amongst the most popular recreational sports activities. Optimizing tennis teaching methods and improving teaching modes can effectively improve the teaching quality of tennis. In this study, a video and image action recognition system based on image processing techniques and Internet of things is developed to overcome the shortcomings of the traditional tennis teaching methods. To validate its performance, the students of tennis courses are divided into experimental group and control group, respectively. The control group is taught by using the traditional tennis teaching method whereas the experimental group is taught by using the IoT video and image recognition teaching system. Three factors of students including service throwing height, arm elbow angle, and knee bending angles of both groups are measured and compared with those of world elite tennis players. The results show that the students' serving abilities in the experimental group are significantly improved using the video and image recognition system based on IoT, and they are better than those of the students in the control group. The proposed video and image processing technique can be applied in students' physical education and can be employed to provide the basis for the innovation of tennis teaching strategies in physical education.

## 1. Introduction

Tennis, as a sport that has a history of over 130 years, is now gaining popularity among ordinary people. Tennis is an Olympic sport and is played at all levels of society and all ages. Tennis is a sport that not only provides a full-body workout but also helps students become sharper and more alert, thereby improving academic performance [1]. At present, the traditional teaching methods are still used in tennis teaching in colleges and universities, which seriously affects the progress of tennis in colleges and universities. In traditional tennis teaching, after understanding the basic contents, students can learn skilled technical actions through repetitive mechanical exercises. Traditional tennis teaching methods stress basic knowledge and elementary technical tennis movements, disregarding students' learning experience. Traditional tennis teaching mainly includes warm-up activities, descriptions of teachers' technical movements, and frequent exercises [2]. In addition, the traditional teaching method of teacher demonstration and student imitation is outdated and cannot meet the requirements of society, making students have difficulty in understanding the key points of tennis playing thoroughly. Therefore, a new tennis teaching strategy is needed to overcome the traditional teaching method [3].

In tennis teaching, the tennis serving process can be regarded as receiving badminton. However, the difficulty of tennis teaching lies in how to teach students to serve tennis correctly [4]. Hayes et al. [5] thought that an individual's thigh strength, body coordination, and upper limb strength have different effects on the serving posture. Fett et al. [6] found that the angle between the tennis ball and the reference line affects the service efficiency. Jiang and He [7] proved that shoulder training can improve tennis service efficiency. In addition to personal physical elements, Kocib et al. [8] summarized that in tennis doubles, the position of players in the team and the type of formation affect the standard degree of service. This shows that teaching students to serve a tennis ball correctly is a challenging task [9].

With students' rising interest in sports and physical fitness, tennis is gaining universal attention. Recent tennis well combines speed and strength and has high requirements for players' physical quality and tactics. Using advanced technological approaches, tennis players' main action video images can be collected and analyzed to help improve their skills. Sports actions caught by computer vision systems can be utilized for player detection and tracking, pose estimation, and movement analysis [10]. The mechanism of the computer vision-based sports action recognition is comprised of player's action detection and tracking, cropping, and targeted actions recognition, which depend upon the sport type and vision system [11]. The computer vision-based sports action recognition systems can provide rapid postmatch analysis and real-time objective feedback before the next race for coaches and players. Bera et al. [12] pointed out that the fundamental points of athletes' actions could be captured via three-dimensional video shooting techniques. Yu and Chin [13] recorded athletes' time-spatial action images via radio frequency technology in IoT, which turned out to be blurred and could not be seen clearly. With the advancement of image and video processing, super-resolution reconstruction and deblurring techniques have also achieved considerable development. Zhou et al. [14] applied super-resolution optimization techniques to increase sports image resolution. Pratim Ray [14] explored that sports and recreational activities can be augmented through novel services based on Internet of Things and showed that the data convergence time is directly proportional to the number of players. The authors in [14] used data mining techniques to examine the technical calibration and related parameters in sports and constructed a sports action recognition system. Pratim Ray [15] established a platform of sports behavior mining and personalized health service based on big data analysis framework for mobile medical technology to provide health protection for users.

To sum up, a research hotspot is rising for the collection and optimization of real-time tennis video images to improve players' actions and skills. In this study, a video and image processing technology based on Internet of things (IoT) is used to establish the recognition system for tennis serving, and the degrees of serving standard between the experimental group and the control group in tennis teaching of a university are compared to discuss whether the system is feasible. The proposed system provides the basis for the innovation of tennis teaching strategies in physical education and can help physical education (PE) teachers to carry out their activities.

The rest of the manuscript is ordered as follows: Section 2 describes the proposed research method in detail. In Section 3, the results are illustrated, and a comparative analysis is provided between the control and experimental group. The conclusion is given in Section 4.

## 2. Materials and Methods

### 2.1. Concept of IoT Video and Image Processing Technique

IoT and image processing have been so far been used for various applications independently. Their application in the field of industries exists and has achieved a certain degree of success. IoT is widely used in remote antitheft, highway nonstop charging, intelligent library, and remote power meter reading, which promote the application of IoT in other fields. Based on IoT, the intelligent development of transportation, security, monitoring, and logistics, and intelligent control of household appliances are realized through the huge network connected with different objects [16]. However, there are still many problems to be solved in expanding the application of IoT because it is a product that appeared in the development of information technology. In this case, some policies, economic and technological environments, microsensors, UHF chips, cloud computing, and information security are ready to support the development of IoT. The video and image processing technique is to process videos and images by using IoT data, including software processing of multimedia files, and the development and application of software and hardware. At present, most of the image processing technologies are multiple processing technologies based on computer technology platforms [17], through image shooting, collection, and compression, coding, and editing. The earliest technology for video processing was in the 2D space.

At the end of the 20th century, video application technology is developed in 3D space [14] and gradually integrated into human life [18]. Today's video processing technology has gradually developed into an emerging industry.  Figure 1 shows the three-tier process of video processing, which includes video or image processing, analysis, and understanding.  Table 1 shows the terms often used in video processing [15]. Using these terms, a comprehensive understanding of video processing is realized.

In multimedia video processing, the following terms are frequently used.

  Frames: it is the number of frames is presented per second, and it shows the updating times of the image processing scene per second. The more the frames are, the smoother and clearer the image will be. Generally, 30 frames are acceptable. If the frame rate exceeds the screen refresh rate, it will waste the energy of the image processor.
  Image Refresh Rate: it refers to the refresh times of the screen per second. The refresh rate is divided into the vertical refresh rate and the horizontal refresh rate. Generally, the vertical refresh rate is used. The vertical refresh rate shows the times the image is redrawn on the screen per second, that is, the times the screen is refreshed per second. The higher the refresh rate is, the more stable the image is and the more natural and clear the image is. On the contrary, if the refresh rate is low, the image will flash greatly, which is harmful to human eyes [19]. The flash screen can be avoided when the refresh rate is above 80 Hz.
  Screen Resolution: it refers to the size of the image formed by video imaging products
  Video Bit Rate: it is the bit rate. It refers to the number of bits playing continuous media (such as compressed audio and video) per unit of time. The higher the bit rate is, the more bandwidth will be consumed. The bits are either 0 or 1.

In this study, multiple IoT video image processing techniques are used to accomplish the experiment.  Figure 2 shows the roadmap of multivideo and image processing technology. The videos are collected and stored on the site without interference, which is the basis of video and image processing. Next, different kinds of processing methods are used to evaluate the posture of the players in specific sports. The principles and processes of video and image processing are diverse. The task of analyzing students' movement and posture can be achieved only by applying the specific image and video processing technique [20].  Figure 3 illustrates the structure of the fast-processing feedback system, which includes equipment for video collection, video transmission and storage, processing, and display methods, forming a complete processing chain.

The video collection process involves a variety of devices, and the collection methods are also diversified. According to different usages and research directions [21], the video collection methods are also different.  Figure 4 shows the hardware requirements and some common collection methods of videos.

Because of different research purposes, different processing methods are required. The general image processing methods are cutting, decomposition or synthesis, zooming in and out, moving, rendering, and adding or dubbing texts [22].  Figure 5 shows the common video and image processing methods in the field of sports.

### 2.2. Colour Processing in Video Image Processing

The perception of color is of supreme importance in many applications, such as digital imaging, multimedia systems, computer vision, entertainment, and consumer electronics. Colour has been becoming a vital element for many, if not all, current image and video processing systems. Colour plays a dominant role in digital photography systems such as digital cameras, video displays, video-enabled cellular phones, and printing solutions. In color image processing, an abstract mathematical model known as color space is used to describe the colors in terms of intensity values. In this color space, a three-dimensional coordinate system is used. For different types of applications, several different color spaces exist.  Figure 6 shows that there are three primary colors in nature, namely red, green, and blue (RGB). Other colors are obtained by mixing the three primary colors in different proportions [23], and the three primary colors can be overlapped to obtain pink, cyan, yellow, and white. The advantage of RGB is that they are simple to understand and easy to distinguish. Trichromatic RGB is a color space that depends on the detection and reproduction of the RGB values by different equipment and is different because the color substances (fluorescent agents or dyes) and their response levels to red, green, and blue vary with different manufacturers. The three primary colors are red, green, and blue, and their corresponding wavelengths are 700 nm, 546.1 nm, and 435.8 nm, respectively, and they are different from those of the object. The three primary colors, when mixed in a certain proportion, can present various light colors. According to the research results, the three primary colors are determined as red, green, and blue (equivalent to the color feeling of bright red, medium green, and ultramarine).

The color discrimination algorithm is based on colorimetry. *r*, g, and *b*, respectively, represent the proportion of the stimulus value of the three primary colors in the total RGB, and R, G, and B, respectively, represent the chromaticity coordinates of the chromaticity system. The chromaticity of another color is jointly determined by R, G, and B. The equations are as follows:

(1) $$\begin{array}{c} r=\frac{R}{R+G+B},\\ g=\frac{G}{R+G+B},\\ b=\frac{B}{R+G+B},\\ r+g+b=1. \end{array}$$

If *r*, g, and *b* represent three-pixel value channels of the input video or image, the value range is usually [0, 255]. The three channels are nonlinear and need to be corrected. They are computed as follows:

(2) $$\begin{array}{c} R=\text{gamma}\left(\frac{r}{225.0}\right), \end{array}$$

(3) $$\begin{array}{c} G=\text{gamma}\left(\frac{g}{225.0}\right), \end{array}$$

(4) $$\begin{array}{c} B=\text{gamma}\left(\frac{b}{225.0}\right), \end{array}$$

(5) $$\begin{array}{c} \text{gamma}\left(x\right)={\left(\frac{x+0.055}{1.055}\right)}^{2.4},\;\;x＞0.4045, \end{array}$$

(6) $$\begin{array}{c} \text{gamma}\left(x\right)=\left(\frac{x}{12.92}\right),\text{other}. \end{array}$$

Since there are color blind individuals in the population, it is necessary to optimize the system and incorporate the color blindness correction.  Figure 6 shows a two-color vision process in which the system calculates and replaces ordinary colors to meet the color recognition standard of color-blind individuals. The color gamut needs to be adjusted and scaled appropriately to make the mapped color within the realistic color range of the device. For example, for red blind individuals, the following adjustments are made:

(7) $$\begin{array}{c} R_{2}=0.992052R+0.003974,\\ G_{2}=0.992052G+0.003974,\\ B_{2}=0.992052B+0.003974. \end{array}$$

For individuals with green blindness, the following adjustments need to be made:

(8) $$\begin{array}{c} R_{2}=0.957237R+0.0213814,\\ G_{2}=0.957237G+0.0213814,\\ B_{2}=0.957237B+0.0213814. \end{array}$$

Using the color correction process given in equations (2)–(6), the color value of color blind individuals can be obtained.

### 2.3. Evaluation of Action Standard of Tennis Service

The serve in tennis is usually considered the most significant stroke in the game because it is a high predictor of match success, with its effectiveness primarily dependent on ball speed.

The service process of tennis can be ordered as being calm, stabilizing the racket, preparing to serve, throwing the ball, powerful swing, and hitting the ball. The tennis service can be divided into three types: flat serve, cutting services, and topspin (kick) serve. Each kind of service has its characteristics and advantages. A good serve is powerful, and the speed, power, rotation, and landing point of the ball are different from the expected. Flat serve is the fastest among all kinds of services, and its speed is fast and cannot rebound. Cutting serve is a service method based on right rotation (slightly downward rotation). Because of the flight track and bouncing direction, it is fast and threatening, and the service hit rate is improved. It is adopted by most athletes all over the world. Topspin serve is a service method dominated by topspin and supplemented by lateral spin. Because the upward rotation of the ball is more than that of the cutting serve, the ball produces an obvious arc flight path from top to bottom. The stronger the force is, the more the rotation component is, the larger the arc is, and the higher the hit rate is. The ball will land on the left of the other party, forcing the rival to receive the ball from the position and causing great pressure on the opponent.

In this study, the students who attended the tennis course were categorized as the experimental subjects, and all the students were divided into the experimental group and the control group. The experimental group is taught with the help of the proposed tennis serve action recognition system, and the control group is taught by the traditional teaching method, as shown in Figure 7.

The traditional teaching method used by the control group is shown in Figure 8. This method of teaching mainly focuses on skill teaching. Through teacher demonstration and students' imitation, they passively receive knowledge and repeat the same practice. Next, the teacher corrects the actions of the students, and the students imitate the teachers' actions again. After the serving posture is measured, the arm angle and the serving height of the throwing ball are used as the reference data for comparison.

The experimental group used the IoT video and image recognition technique to carry out the teaching activities, as shown in Figure 9. First, through the key points explained by the teacher, the students were shown the videos of the service actions of excellent tennis players to enable the students to accomplish correct tennis actions. Second, the recognition system was used to shoot and identify the students' service actions, and the shot video was used to analyze the throwing height of the service and the angle of the arm joint.

Finally, appropriate standardized teaching tasks were designed, and their correct service postures were referred to make error corrections for students. The work was repeated every day to complete the service training task. In this experiment, several principles are followed which are shown in Table 2.

To determine the feasibility of the video image recognition system, the method is evaluated using the serving data of the world's famous tennis players.  Table 3 shows the data of the relative angle between the throwing height of the world's famous players and their arms and knees.

During the experiment, the above three kinds of data are measured when students served the tennis balls, and the experimental results of the experimental group and the control group are compared to judge whether the proposed video image recognition system can be applied in tennis serving teaching.

## 3. Results

### 3.1. Comparative Analysis of Students' Movements and Postures in Tennis Serving Teaching

The tennis serve is the most difficult stroke in competitive tennis. The complexity of the actions results from the combination of the upper and lower limb and joint movements essential to combine and transfer forces from the ground up through the kinetic chain and out into the ball. Active servers excellently utilize their full kinetic chain through the simultaneous application of selective muscle groups, segmental rotations, and coordinated lower limb muscle actions (hamstrings, quadriceps, and hip rotators). This lower extremity core force is then transferred up into the upper extremity and out through the racket into the ball. If any of the links in this chain are not synchronized efficiently, the result of the serve will not be optimal. To evaluate the proposed tennis serving method, the tennis service action data of the experimental group and the control group are recorded and compared, respectively. The recorded data are the throwing height during service, the arm elbow angle of clapping hands, and the bending angle of the knee joint. After the experiment, the average value of the data of the two groups is compared. The data recorded are shown in Figure 10.

In Figure 10, the first two histograms correspond to the experimental group and the control group, respectively, and the third histogram shows the serve data of famous tennis players as the basis for comparison.

It is evident that the results of the experimental group are closer to those of the 'world's elite tennis players in terms of the throwing height of the service, the angle of the arm and elbow, and the bending of the knee joint. In the experimental group, the results obtained for throwing height of the service, the angle of the arm and elbow, and the bending of the knee joint are 119.6 m, 72.18°, and 3.8°, respectively. The results of the control group are quite different from the results of the elite players, with the difference in the throwing height of about 0.77 M, that is, the relative angle of the arm and elbow is 12.7°, and the difference in the bending angle of the knee joint is 16.4°, which is larger than the difference results of the experimental group and world's elite players. Therefore, from the comparative analysis of tennis service in three groups, the following conclusions are drawn: the experimental group is taught by the established video and image recognition system as the teaching method of tennis service, and their data gradually approach the service data of the world's excellent tennis players. This shows that the proposed teaching method significantly improves the tennis serving level of the students in the experimental group. This shows that the image processing technique can greatly promote the development of the theory and practice of tennis training and optimization. Tennis training must take full advantage of proposed video and image processing techniques according to their characteristics to improve the quality of tennis training and improve the quality of athletes. Furthermore, this video image analysis technique comprehensively applies the image data synthesis technique to realize the real-time analysis of tennis tactics and simultaneously outputs the analysis results.

## 4. Conclusions

Tennis training analysis based on image and video processing is a research hotspot and complex point in computer vision. It predicts moving objects from image and video sequences, extracts prominent parts of the human body, and obtains useful information for human movements to obtain human action and postures. Because of the incompetent teaching ability and the outdated teaching mode of teacher demonstration and student imitation in tennis, a video image action recognition system is proposed based on IoT. It is established based on the video and image analysis techniques and the ability of color discrimination and applied to the teaching of students' tennis service action correction. The students of tennis courses are divided into the experimental group and the control group. The experimental group is taught by using the IoT video and image recognition teaching system and the control group is taught by using the traditional teaching method. The results of tennis service actions of both groups are compared with the results of world elite tennis players. It is found that the service level of students using the proposed method is significantly improved and better than that of students in the control group. Therefore, it is concluded that this action recognition teaching system based on a video image can be applied to students' tennis teaching and can also be deployed in other sports.

## Figures and Tables

**Figure 1:** Three-tier process of video and image processing.

**Figure 2:** Roadmap of multivideo and image processing technology.

**Figure 3:** Structure of the fast-processing feedback system.

**Figure 4:** Collection devices and collection methods.

**Figure 5:** The simple flow of video and image processing in sports.

**Figure 6:** Simulation coordinates of other colors.

**Figure 7:** Experimental image collection site.

**Figure 8:** Traditional teaching methods used in the control group.

**Figure 9:** Teaching methods adopted by the experimental group.

**Figure 10:** Comparison results of tennis serve actions.

**Table 1:** Common technical terms of video and image processing.

Terms	Components
Video production	NTSC (National Television System Committee) and PAL (phase alternating line) are widely used in American countries (30 frames/s), while the latter is widely used in China (25 frames/s)
Resolution	It includes the concepts of the pixel, image resolution, and display resolution. The smaller the pixel size is, the more pixels in the same display there are, and the clearer the video or image is
Image format	Generally, there are BMP, JPG, tiff, PCX, and GIF. Because the storage space of current digital cameras is small, the images are generally transmitted to the computer for storage
Video format	There are many kinds of video formats, their compression and coding methods are different, and they need to be converted frequently. The commonly used formats include MP4, AVI, and MPEG [17]
Types of videotapes	Normal photographing can only be carried out when the videotape corresponds to each camera and the photographing equipment
Video and image processing medium	The optical discs (DVD and VCD) are used for storage in earlier times, and now you can store video in digital format on the computer
Video capture card	The function of the capture card is to transmit video or image to the computer and save it in the format of the data file. It is an indispensable technology for video and image processing

**Table 2:** Experimental principles.

Experimental principles	Specific meanings
Scientific principle	According to this principle, experimental materials, the methods, the selected subjects, and the processing method of the results must be scientific. In terms of experimental subjects, it is ensured that the number of experimental group and control group is the same, and the experiment should be carried out secretly
Comparative principle	It means that the image processing system is used in the tennis serving course. The experimental process should not be affected by other factors. The influence of objective factors shall be eliminated as far as possible in the experimental process. Moreover, it is ensured that the number of subjects, places, equipment, and course content is consistent with the course time
Control single variable	The variable to be controlled in this experiment is the teaching method. This means that the experimental group can only use the video image processing and recognition system, and the control group can only use the traditional teaching method, which are the most basic and important conditions in the experiment. Whether the experimental results are persuasive depends on the principle of controlling a single variable

**Table 3:** Serving data of famous tennis players.

Evaluation standards	Throw height of serving (m)	Arm elbow angle of clapping hands (°)	Bending angle of knee joint (°)
Evaluation value	3.9	72.55	116.5

## Data Availability

The data used to support the findings of this study are included in the article.
